# Reduced levels of A20 protein prompted RIPK1-dependent apoptosis and blood–brain barrier breakdown during cerebral ischemia reperfusion injury

**DOI:** 10.1371/journal.pone.0290015

**Published:** 2023-08-14

**Authors:** Chaonan Yang, Yongjiao Wang, Xiaohui Wu, Min Gong, Ying Li

**Affiliations:** 1 Department of Pharmacy, Tianjin Medical University, Tianjin, China; 2 WIMM, University of Oxford, Oxford, United Kingdom; 3 Tianjin Neurological Institute, Tianjin Medical University General Hospital, Tianjin, China; Lady Hardinge Medical College, INDIA

## Abstract

Blood–brain barrier (BBB) leakage is an important cause of the exacerbation of pathological features of cerebral ischemia reperfusion injury (CIRI). However, the specific mechanism of BBB leakage is not clear. It was found that the CIRI resulted in RIPK1 activation and subsequent RIPK1-dependent apoptosis (RDA). Inhibition of RIPK1 significantly reduced BBB breakdown and brain damage. The aim of this study is to investigate the mechanism of RIPK1 in the BBB leakage during CIRI. It was discovered by proteomics that autophagy activation resulting from ischemia and reperfusion significantly downregulated the level of A20 protein. A20 is an important protein that regulates RIPK1 and RDA. It was hypothesized that activation of autophagy caused by ischemic reperfusion led to a decrease in A20 protein, which, in turn, caused the activation of RIPK1 and the occurrence of RDA, leading to leakage of the BBB. The findings in this study revealed the role of RIPK1 in the cell death and BBB leakage upon cerebral ischemia reperfusion injury, and these findings provide a novel perspective for the treatment of ischemic reperfusion.

## Introduction

The BBB is an anatomical and biochemical barrier that protects the brain from potentially harmful substances [1]. The BBB is a highly selective membrane barrier in the brain microvasculature that facilitates transport between the systemic circulation and the central nervous system [2]. The BBB regulates homeostasis of the central nervous system (CNS) by forming a tightly regulated neurovascular unit (NVU) that includes endothelial cells (ECs), pericytes and astrocytic endfeet, which jointly maintain normal brain function [3–5]. The presence of the BBB is capable of preventing some substances, mostly harmful, from entering the brain tissue from blood. The BBB acts as a physical and metabolic barrier between the CNS and the peripheral circulation, exerting regulatory and protective effects on the microenvironment of the brain [6]. Under normal circumstances, the primary function of the BBB is to establish and maintain homeostasis in the CNS. Once the BBB is destroyed, the brain is particularly vulnerable to infection and damage [7–9].

CIRI remains a leading cause of disability and death globally, and its therapeutic management is an extremely challenging problem in clinical practice [10]. The recovery of blood supply, referred to as reperfusion, has been considered a standard therapeutic option for ischemia [11]. In addition to preventing the growth of infarction volume, reperfusion has been reported to aggravate ischemic damage, including early disruption of the BBB [12–14]. One of the pathophysiological characteristics of CIRI is the destruction of the BBB [13]. During CIRI, BBB damage leads to the infiltration of inflammatory cells into the brain, which further aggravates cerebral inflammation and edema [15–17]. Thus, increasing attention is turning towards the identification of potential targeted drugs to protect the BBB against ischemia–reperfusion injury.

CIRI can result in brain microvasculature and BBB breakdown, leading to increased BBB permeability [18, 19]. Disruption of the BBB following CIRI results in brain edema, a primary event that affects both morbidity and mortality [20]. Subsequently, various mediators are released that enhance vasogenic and/or cytotoxic brain edema [21]. These include glutamate, lactate, H^+^, K^+^, Ca^2+^, nitric oxide, arachidonic acid and its metabolites, free oxygen radicals, histamine, and kinins [21]. The permeability of the BBB to endogenous proteins, such as immunoglobulin G (IgG), is increased following experimental CIRI [22, 23]. An additional consequence of BBB disruption is the infiltration of leukocytes into brain tissue, accompanied by microglial activation and inflammation [22].

Brain microvascular ECs are a key component in the pathophysiological mechanism of BBB dysfunction after ischemic reperfusion. However, the regulatory mechanism governing endothelial cell death is still unclear. Recently, it was implied that Receptor Interacting Protein Kinase 1 (RIPK1), which is a crucial necroptotic and apoptotic mediator in CIRI, might play an essential role in regulating endothelial cell death during the progression of CIRI [24–26]. RIPK1 is a serine/threonine protein kinase. The kinase activity of RIPK1 is stimulated by the tumor necrosis factor-α (TNF-α) death signal, and subsequent downstream necroptosis is activated [27]. Necroptosis, a form of regulated necrosis, is a caspase-independent regulated type of cell death pathway which is mainly composed of the RIPK1, receptor-interacting protein kinase-3 (RIPK3) and mixed lineage kinase domain-like protein (MLKL) [28, 29]. Activated RIPK1 self-phosphorylates at serine 166, then recruits RIPK3 and MLKL [30, 31]. The polymer RIPK1/RIPK3/MLKL leads to cell necroptosis during the progression of CIRI [32–34]. Necrostatin-1 (Nec-1/Nec-1s), the small-molecule inhibitor against necroptosis, resulted in significant reduced infarct volume in MCAO mice [29]. Necrostatin-1 was then found to be a highly specific inhibitor of RIPK1 kinase which remarkably retarded the necroptotic damage to neurons [35]. Except the necroptosis induced by RIPK1, it was convinced that the activation of RIPK1 also mediated a special apoptotic cell death pathway by forming complex with FADD and caspase-8 under apoptosis-proficient conditions in CIRI [36, 37]. In contrast, under the apoptotic-deficient condition such as the presence of caspase inhibitor, TNF-α promotes the activation of RIPK1 and leads to RIPK1/RIPK3/MLKL necroptotic pathway [38]. However, the physiological mechanism of RIPK1 in the interchange between necroptosis and apoptosis are unknown, which was presumed to be essential for demonstrating the pathogenesis in CIRI damage. The *Ripk1*^D138N^ mutant mice were employed in this study since D138N mutant resulted in the inactivation of necroptosis, however, the *Ripk3*^-/-^ KO mice were employed as necroptosis deficient model. The selection of model animals aimed to clarify the physiological role of apoptosis and necroptosis during the cerebral ischemia reperfusion injury.

In this study, the physiological function of RIPK1 was investigated to elucidate the mechanism of BBB destruction during the process of CIRI, which might contribute to the development or optimization of a clinical intervention approach.

## Materials and methods

### Antibodies and reagents

The following antibodies were employed: mouse anti-MLKL (Abcam), mouse anti-caspase 3 (Cell Signaling), mouse anti-cleaved caspase 3 (Cell Signaling), mouse anti-pRIPK1(S166) (Lifespan) and mouse anti-pMLKL(S345) (Novus). Secondary horseradish peroxidase HRP-conjugated antibodies were from Abcam.

### Mice and treatments

The pathogen-free male wild-type C57BL/6J mice (n = 24), *Ripk1*^D138N^ mice (n = 3) (on a C57BL/6J background) and *Ripk3*^-/-^ mice (n = 3) (on a C57BL/6J background), 8 to 11 weeks of age, were provided by Model Organisms (Shanghai, China). Animal experiments were carried out in accordance with ARRIVE guidelines and of the China Animal Care and Use Committee of Tianjin Medical University (Application Number 201910017).

The animals underwent the middle cerebral artery occlusion (MCAO) procedure to construct a CIRI model. Mice were injected with 3% pentobarbital sodium (80 mg/kg) intraperitoneally. The common carotid artery, internal carotid artery and external carotid artery were separated after the skin of the head was prepared and disinfected. Then, briefly, a monofilament (0.18 mm) was introduced into the common carotid artery under anesthesia, advanced to the origin of the MCA, and left there for 2 hours. After 2 hours of ischemia, the filament was pulled out to enable reperfusion, and the skin was sutured. The mice were placed on a heating pad and then transferred to an incubator after waking up. The brains of anesthetized mice were removed at 1 h, 6 h, 12 h, 24 h and 48 h after reperfusion for further experiments. Sham operations were performed following the same procedure, except that the surgery was stopped after the dura mater was opened.

### shRNA design, cloning, and viral vector construction

siRNA sequences against A20 (NM_001270507) were designed using an online algorithm (http://sidirect2.rnai.jp) (5′-AGTTTCAACCGTCTTAATCAG-3′, 5′-GATTAAGACGGTTGAAACTAG-3′). The indicated sequences were cloned downstream of a human Cdh5 promoter in a pAAV2-CMV-GFP vector provided by the Tianjin Institute of Pharmaceutical Research. A recombinant virus was produced by the Vector Builder (Tianjin Institute of Pharmaceutical Research) using a baculovirus system, and virus titer is 10^12^ V.G./ml. In the A20 knockdown experiment, a total volume of 15 μl viral vector suspension was injected into tail vein of C57BL/6J mice (AAV-shCtrl group n = 26 mice, AAV-shA20 group n = 14 mice). After injection, 14 days were needed for successful transfection before MCAO treatment.

### TTC staining

Wild-type, *Ripk1*^D138N/D138N^ and *Ripk3*^-/-^ mice were deeply anesthetized with sodium pentobarbital (80 mg/kg). The brains were removed quickly (within 10 min) and transferred into a -20°C refrigerator for 30 min, after which coronal brain sections (2 mm thickness) were stained with 2% red tetrazolium solution (Sigma-Aldrich, USA) for 30 min at 37°C in the dark. The container was slightly shaken every 5 min to ensure full staining. The brain slices were washed with PBS solution for 3–5 min and then fixed with 10% neutral formaldehyde for 6 hours, after which images were captured immediately.

### Immunofluorescence (IF)

The whole brains of wild-type, *Ripk1*^D138N/D138N^ and *Ripk3*^-/-^ model mice those after MCAO/R treatment were removed after various periods of reperfusion (1, 6, 12, 24 or 48 hours). The whole brains were fixed in 4% paraformaldehyde solution for 48 h and then sliced into 3- to 5-μm sections on the slides after being embedded in paraffin. Following deparaffinization, the sections (3–5 μm thick) on slides were subjected to high pressure and heat in citrate buffer solution (pH 6.0, 0.01 M, 1000 ml; Abcam, UK) for 2 min for antigen retrieval. The samples were incubated in 3% H_2_O_2_ at room temperature for 4 min and then blocked with 10% BSA at room temperature for 30 min. The ischemic cores were employed for immunohistochemical assays.

The activation of p-RIPK1 (S166) and cleaved caspase 3 (CC3) in mice treated with MCAO/R was detected by immunofluorescence using DAPI staining according to the manufacturer’s instructions. CD31 was measured as an indicator of endothelial cells, and PI staining was employed to detect apoptosis. IgG was detected in this study to evaluate BBB permeability. The slides were observed using a fluorescence microscope (BX51; Olympus Corporation, Tokyo, Japan).

### Immunoblotting

The brain tissues of treated mice were collected at 1, 6, 12, 24 and 48 hours after cerebral ischemia and reperfusion. The tissues were ground, and their protein levels were measured by Western blotting. Aliquots of protein extracts were subjected to 12% SDS-PAGE. After electrophoresis, the proteins were transferred to a PVDF membrane (Amersham Biosciences) and then incubated with the desired primary antibodies (anti-A20 and anti-CC3) and secondary antibodies according to the manufacturer’s instructions. Finally, the proteins were detected with Luminol ECL reagent (Thermo Scientific). Densitometry was performed using ImageJ software. All gels and densitometry shown are representative of at least three experiments unless otherwise indicated.

### Statistical analyses

Data are expressed as the mean ± SEM. Significance was assessed with Student’s t-test or one-way ANOVA followed by Bonferroni’s post hoc test using Prism version 6.0 software (GraphPad). P values below 0.05 were considered significant.

## Results

After MCAO treatment, the *Ripk1*^D138N^ mice showed remarkable ameliorating infarction area but *Ripk3* knock out mice did not (Fig 1A). The finding ascertained that RDA played dominant role in the infarction instead of RIPK-1 associated necroptosis [39]. In this study, the activation of RIPK1 protein was investigated upon the phosphorylation-serine 166 [40] by western blotting (in Fig 1B and 1C). Result exhibited the wild-type and *Ripk1*^D138N^ mice showed significant increase in the phosphorylated level of RIPK1(S166) but not the *Ripk3*^-/-^ mice. The p-RIPK1 level was only increased 24 hours after MCAO treatment in *Ripk3* knock out mice. This finding ascertained that the dead knockin allele D138N in RIPK1 is crucial for kinase activation which was contributed to the infarction volume.

**Fig 1:** Analysis of phosphorylation of RIPK1 by ischemic insult. **(A).** The WT, *Ripk1*^D138N^, and *Ripk3*^−/−^ mice were subjected to transient 90-min MCAO, followed by reperfusion. The brains of mice were processed for TTC staining to measure infarct volume (n = 11 per group). **(B) and (C).** Brain lysates from mice with indicated genotypes subjected to MCAO for 90 min followed by reperfusion for the indicated time periods were analyzed by immunoblotting with p-S166 RIPK1 antibodies. The data in (A) indicated that the infarcted size after CIRI in mutant *Ripk1*^D138N^ mice was significantly smaller than that in wild-type mice but not the *Ripk3*^-/-^ mice. The finding indicated the crucial physiological role of RDA in the infarcted formation. (B) and (C) showed significant increase in the phosphorylated level of RIPK1(S166) in *Ripk1*^D138N^ mice but not the *Ripk3*^-/-^ mice. This finding ascertained that the dead knockin allele D138N in RIPK1 is crucial for kinase activation which was contributed to the infarction volume.

In order to evaluate the permeability of the BBB during the process of ischemia and reperfusion, the penetration of immunoglobulin G (IgG), an endogenous protein, was monitored. An immunofluorescence assay indicated that IgG penetration was significantly increased 3 days after ischemia and reperfusion, suggesting the destruction of the BBB following the stimuli associated with CIRI (Fig 2). Moreover, the permeability of the BBB was remarkably weakened in *Ripk1*^D138N^ mutant mice, which inhibited RIPK1 activation after MCAO procedure (Fig 2). These results demonstrated that RIPK1 activation may play an important role in BBB destruction.

**Fig 2:** Inhibition of RIPK1 activity retarded BBB leakage. (A). The measurement of permeability of the BBB in wild-type and *Ripk1*^D138N^ mutant mice. (B). The quantifications of fluorescence intensity of p-RIPK1 and leaked IgG during CIRI. After the MCAO/R experiment (3 days), the penetration of IgG in the brain was measured to evaluate BBB permeability. The BBB was destroyed in wild-type mice (n = 5) after MCAO treatment; however, it showed significantly increased tolerance to CIRI in *Ripk1*^D138N^ mutant mice (n = 3). (* represent *p*<0.05 and ** represent *p*<0.01).

RIPK1 was activated to a remarkable extent in cells upon the occurrence of CIRI, and a series of MCAO animal experiments and immunofluorescence assays were performed to clarify whether RIPK1-induced BBB destruction was RIPK3 dependent. TTC staining data showed that the volume of cerebral infarction in *Ripk3* gene knockout mice remained similar to that of wild-type mice; however, the *Ripk1*^D138N^ mutant mice showed a significantly reduced volume of post-MCAO cerebral infarction (Fig 3B).

**Fig 3:** MCAO in RIPK3 knockout mice (*Ripk3*^-/-^). **(A).** Apoptosis in various mice upon MCAO treatment. Images show the results of CD31 (green) and PI (red) staining in brain sections from MCAO-treated mice. The results indicated that *Ripk3* knockout (n = 3) only partially inhibited cell death, in contrast to *Ripk1*^D138N^ (n = 3). (Animals employed in shammed and control group was 6, respectively). **(B).** Effect of RIPK3 knockout on cerebral infarction volume. After MCAO/R, the brains of mice (n = 4) were sectioned and stained with TTC. The infarct volume of mouse brains after TTC staining was quantified (n = 27). The results showed that *Ripk3* gene knockout did not reduce the volume of cerebral infarction as *Ripk1* mutation did (*Ripk1*^D138N^ in Fig 1), suggesting that RIPK3 may play a limited role in CIRI. **(C). Analysis of apoptosis activity effected by** RIPK3. The level of cleaved caspase 3 (CC3) in the cells of *Ripk1*^D138N^ mice was significantly decreased; however, the protein level of CC3 was maintained in *Ripk3*^-/-^ mice. The results suggested that the apoptosis in ischemic reperfusion injury is mainly caused by RIPK1-activated apoptosis rather than programmed necrosis.

Furthermore, the death of cells in MCAO experimental mice was assessed by PI staining. The results showed that *Ripk3* knockout did not inhibit cell death as effectively as *Ripk1*^D138N^ but achieved only partial inhibition (Fig 3A), suggesting that RIPK3 may play a limited role in ischemia-reperfusion injury. Considering that RIPK3 was associated only with RIPK1-mediated necroptosis in CIRI, it was presumed that RIPK1-mediated programmed cell necrosis might not be the main cause of cell death in the BBB upon ischemia and reperfusion stimuli. Subsequently, it was speculated that RIPK1-dependent apoptosis (RDA), as opposed to RIPK1-mediated necroptosis, might play a dominant role in the leakage of BBB.

The apoptosis marker cleaved caspase 3 (CC3) was employed in this study to evaluate the effect of RDA on BBB destruction during the progression of ischemia–reperfusion injury [41, 42]. Immunoblotting data showed that an inactive mutant form of RIPK1 (*Ripk1*^D138N^) inhibited the initiation of RDA in mice after MCAO treatment; however, the RDA features remained intact in the *Ripk3*^-/-^ mice (Fig 3C). The results suggested that the cellular death in MCAO mice was caused mainly by apoptosis mediated by RIPK1 activation rather than programmed necrosis.

In order to clarify the molecular mechanism of RDA after MCAO, protein mass spectrometry was performed to analyze the mouse brains treated with MCAO. The analysis of up-regulated and downregulated proteins indicated that A20 protein was significantly downregulated (3-fold) after MCAO (Fig 4A). The protein level of A20 was also measured by Western blot after MCAO treatment. Similarly, the mRNA level of A20 was quantified using PCR following MCAO treatment. The results showed that upon CIRI, the protein level of A20 was significantly reduced, but the mRNA level of A20 was not regulated (Fig 4B and 4C), implying that the decrease in the A20 protein level may be associated in ischemic reperfusion.

**Fig 4:** Investigation of the molecular mechanism of RDA. **(A).** Volcano plot of protein expression in brain samples after MCAO treatment. The volcano plot of protein mass spectrometry showed that protein A20 was significantly downregulated after MCAO. **(B).** Protein level of A20 after MCAO treatment. The results indicated that the protein level of A20 was remarkably downregulated after MCAO treatment. After two hours of MCAO and different durations of reperfusion, the brain tissue was ground and assessed by Western blotting. **(C).** mRNA level of A20 after MCAO treatment. The results indicated that the mRNA level of A20 was retained during the process of MCAO. After two hours of MCAO and different durations of reperfusion, brain tissues were collected and ground to measure the levels of A20 mRNA using qPCR. The results suggested that the decrease in A20 levels may be the key cause of RDA in cells in ischemia–reperfusion injury.

Subsequently, A20 knockdown mice were constructed on a C57BL/6J background to evaluate the physiological functions of A20 after MCAO treatment. The results showed that the volume of cerebral infarction and the apoptosis of vascular cells were significantly increased in A20 knockdown mice (A20-EKD) during ischemic reperfusion (Fig 5). This finding suggests that the degradation of A20 protein acts an essential feature in the initiation of RDA and might be deeply associated with cell death and BBB destruction in the progression of ischemia–reperfusion injury.

**Fig 5:** A20 knockdown enhanced RIPK1-dependent apoptosis after MCAO treatment. **(A).** Brain tissues of wild-type and A20-EKD mice. The expression of A20 was measured by Western blotting. **(B).** After MCAO/R, the brains of wild-type and A20-EKD knockdown mice were sectioned and stained with TTC. T2-weighted imaging was used to measure the infarct volume (WT, n = 26; A20-EKD, n = 14). **(C).** Different RDA features in wild-type and A20 knockdown mice. CC3 immunofluorescence staining was performed on the brain tissue of mice after 24 hours of MCAO/R. A20 gene knockdown mice (A20-EKD) were constructed by adenovirus transfection (AAV-shA20) (Panel A). The volume of cerebral infarction during ischemia–reperfusion injury was increased in mutant mice (Panel B). In addition, the knockdown of A20 significantly enhanced apoptosis in cells after MCAO treatment. The results suggested that the degradation of A20 protein may be the dominant mediator of RDA.

## Discussion

The BBB is central to the regulation of cerebral microcirculation due to its characteristic barrier properties and transport system. The BBB is principally composed of cerebral micro cells, which form tight junctions together and are interlaced with astrocytes, pericytes, and a basal lamina [43]. These cells possess specialized receptor-mediated transport mechanisms and barrier properties and contribute equally to the local control of cerebral microcirculation.

CIRI can result in breakdown of the brain microvasculature and BBB, leading to increased BBB permeability [18]. CIRI results in brain edema, a primary event that affects both morbidity and mortality following CIRI. Edema increases intracerebral pressure (ICP) and leads to secondary ischemic injuries by impairing cerebral perfusion and oxygenation [44]. An additional consequence of BBB disruption is the infiltration of leukocytes into brain tissue, accompanied by microglial activation and inflammation [45]. BBB injury is recognized to play an important role in brain injury caused by ischemic reperfusion. Inhibition of BBB destruction and vascular endothelial cell death can greatly ameliorate brain injury [46]. At present, the mechanism of endothelial cell death induced by ischemia and reperfusion injury is not completely clear.

It was found in this study that the activation of the kinase RIPK1 played an important role in CIRI, and the CIRI was significantly ameliorated in kinase-deficient mutant *Ripk1*^D138N^ mice. In addition to the effect on neuronal cell death, the activation of RIPK1 was also associated with cell death, suggesting that RIPK1 potentially features in the physiology of BBB destruction in CIRI. BBB permeability was investigated as an indicator of barrier breakdown in this study. The results indicated the crucial role of RIPK1 activation in BBB destruction upon MCAO treatment. The data showed that wild-type *Ripk1*^+/+^ mice exhibited extensive post-MCAO BBB compared to *Ripk1*^D138N^ mutant mice. These observations imply that RIPK1 activation may play an important role in BBB destruction.

RIPK1 not only relates to necroptosis in which RIPK3 is recruited but also mediates RDA in which caspase is activated. RIPK3 knockout mice (*Ripk3*^-/-^) were employed in this study, and the TTC staining results indicated that *Ripk3* gene knockout failed to ameliorate brain injury after MCAO treatment. Interestingly, RIPK1 was found to be activated in *Ripk3*^-/-^ mice as detected by PI staining after MCAO treatment, suggesting that necroptosis induced by RIPK1 might not be the dominant contributor to endothelial cell death upon MCAO stimulation. Instead, it was speculated that RDA might play a dominant role in endothelial cell death in CIRI. The results indicated that the level of cleaved caspase 3 (CC3) was maintained in endothelial cells of *Ripk3*^-/-^ mice but significantly decreased in *Ripk1*^D138N^ mice. This finding suggested that, instead of necroptosis, the RDA (RIPK1-dependent apoptosis) after CIRI may be the main mechanism of BBB breakdown.

In order to investigate the molecular mechanism of RDA, a proteomic study was carried out. Protein A20 was significantly downregulated (3-fold) after MCAO. Zinc finger protein A20, encoded by the TNFAIP3 gene, possesses deubiquitinase activity [47]. A20 is capable of activating NF-κB and initiating TNFα-mediated apoptosis [47, 48]. Recently, it has been suggested that reducing A20 levels in mouse embryonic fibroblasts can promote RDA and programmed necrosis. Accordingly, the regulatory effect of A20 on RIPK1 activity was investigated in this study. The data showed that the protein level of A20 was decreased by a remarkable degree in MCAO mice, but the mRNA level was maintained. It was speculated that the degradation of A20 protein might be a key cause of cell death in MCAO mice. This hypothesis was tested in A20-EKD mice constructed with an AAV system (AAV-ShA20). The results confirmed that the degradation of A20 may play an essential role in the initiation of RIPK1-dependent apoptosis, resulting in programmed cell death and BBB destruction.

In addition, the proteomic study also revealed that the protein p62, a substrate protein in autophagy, was significantly downregulated in MCAO mice, suggesting the activation of the autophagy system. It was reported that ischemia and reperfusion stimulated both autophagy and the ubiquitin proteasome system, two major intracellular degradation systems. The inhibition of the ubiquitin proteasome system can reduce the progression of ischemia–reperfusion injury, but the effect of its inhibition on autophagy has seldom been studied. It was presumed that inhibiting autophagy in CIRI might help ameliorate the destruction of the BBB.

## Conclusion

The findings in this study demonstrated that the death of cells induced by ischemic reperfusion injury was mediated mainly by the activation of RIPK1. The BBB leakage and infarct volume of RIPK1 mutant mice (*Ripk1*^D138N^) were significantly reduced compared to those of wild-type mice. RIPK1 is the main protein that mediates necroptosis; however, it was found that mice without the capacity for necroptosis (*Ripk3*^-/-^) did not show the same high survival rate as RIPK1 kinase mutant mice (*Ripk1*^D138N^). Additionally, the death of cells in *Ripk3*^-/-^ mice was not significantly improved, indicating that RIPK1-mediated programmed necrosis was not the main cause of BBB injury.

Further investigations in this study revealed that RDA might be responsible for the endothelial cell death that leads to BBB leakage after MCAO treatment. A20 was decreased during cerebral ischemia–reperfusion injury, and A20 acted as a key regulatory protein that inhibited RIPK1 and RDA. The decrease in A20 may be related to degradation during autophagy, and autophagy is known to be activated by CIRI.

Owing to the crucial physiological functions of the BBB, there is an urgent demand for the development of therapeutic strategies to prevent BBB dysfunction (i.e., provide vascular protection) in CIRI. The autophagy system may undergo a distinct set of regulatory changes in response to CIRI.

## Supporting information

S1 Raw images (DOCX)

## Abbreviations

BBB: blood brain barrier
CIRI: Cerebral Ischemia Reperfusion Injury
DND: Delayed Neuron Death
MCAO: Middle-Cerebral-Artery Occlusion

## References

[1] WrobelJK, ToborekM. Blood-brain Barrier Remodeling during Brain Metastasis Formation. Mol Med. 2016;22:32–40. doi: 10.2119/molmed.2015.00207 26837070PMC5004726

[2] WiranowskaM. Blood-brain barrier and treatment of central nervous system tumors. J Fla Med Assoc. 1992;79(10):707–10. .1460453

[3] LaiCH, KuoKH. The critical component to establish in vitro BBB model: Pericyte. Brain Res Brain Res Rev. 2005;50(2):258–65. doi: 10.1016/j.brainresrev.2005.07.004 .16199092

[4] GoKG. The normal and pathological physiology of brain water. Adv Tech Stand Neurosurg. 1997;23:47–142. doi: 10.1007/978-3-7091-6549-2_2 .9075471

[5] CharlesV, MufsonEJ, FridenPM, BartusRT, KordowerJH. Atrophy of cholinergic basal forebrain neurons following excitotoxic cortical lesions is reversed by intravenous administration of an NGF conjugate. Brain Res. 1996;728(2):193–203. doi: 10.1016/0006-8993(96)00398-8 .8864482

[6] RivestS, LacroixS, VallieresL, NadeauS, ZhangJ, LaflammeN. How the blood talks to the brain parenchyma and the paraventricular nucleus of the hypothalamus during systemic inflammatory and infectious stimuli. Proc Soc Exp Biol Med. 2000;223(1):22–38.1063295810.1046/j.1525-1373.2000.22304.x

[7] PetitoCK, CashKS. Blood-brain barrier abnormalities in the acquired immunodeficiency syndrome: immunohistochemical localization of serum proteins in postmortem brain. Ann Neurol. 1992;32(5):658–66. doi: 10.1002/ana.410320509 .1449246

[8] EralinnaJP, Soilu-HanninenM, RoyttaM, HukkanenV, SalmiAA, SalonenR. Blood-brain barrier breakdown and increased intercellular adhesion molecule (ICAM-1/CD54) expression after Semliki Forest (A7) virus infection facilitates the development of experimental allergic encephalomyelitis. J Neuroimmunol. 1996;66(1–2):103–14. doi: 10.1016/0165-5728(96)00031-8 .8964903

[9] WoodmanSE, BenvenisteEN, NathA, BermanJW. Human immunodeficiency virus type 1 TAT protein induces adhesion molecule expression in astrocytes. J Neurovirol. 1999;5(6):678–84. doi: 10.3109/13550289909021296 .10602408

[10] DegterevA, HuangZ, BoyceM, LiY, JagtapP, MizushimaN, et al. Chemical inhibitor of nonapoptotic cell death with therapeutic potential for ischemic brain injury. Nature chemical biology. 2005;1(2):112–9. doi: 10.1038/nchembio711 .16408008

[11] CuevasP, CarcellerF, Munoz-WilleryI, Gimenez-GallegoG. Intravenous fibroblast growth factor penetrates the blood-brain barrier and protects hippocampal neurons against ischemia-reperfusion injury. Surg Neurol. 1998;49(1):77–83; discussion -4. doi: 10.1016/s0090-3019(97)00193-6 .9428898

[12] AokiT, SumiiT, MoriT, WangX, LoEH. Blood-brain barrier disruption and matrix metalloproteinase-9 expression during reperfusion injury: mechanical versus embolic focal ischemia in spontaneously hypertensive rats. Stroke. 2002;33(11):2711–7. doi: 10.1161/01.str.0000033932.34467.97 .12411666

[13] PlutaR. Blood-brain barrier dysfunction and amyloid precursor protein accumulation in microvascular compartment following ischemia-reperfusion brain injury with 1-year survival. Acta Neurochir Suppl. 2003;86:117–22. doi: 10.1007/978-3-7091-0651-8_26 .14753418

[14] PillaiDR, DittmarMS, BaldaranovD, HeidemannRM, HenningEC, SchuiererG, et al. Cerebral ischemia-reperfusion injury in rats—a 3 T MRI study on biphasic blood-brain barrier opening and the dynamics of edema formation. J Cereb Blood Flow Metab. 2009;29(11):1846–55. doi: 10.1038/jcbfm.2009.106 19654585PMC2848453

[15] WarachS, LatourLL. Evidence of reperfusion injury, exacerbated by thrombolytic therapy, in human focal brain ischemia using a novel imaging marker of early blood-brain barrier disruption. Stroke. 2004;35(11 Suppl 1):2659–61. doi: 10.1161/01.STR.0000144051.32131.09 .15472105

[16] DimitrijevicOB, StamatovicSM, KeepRF, AndjelkovicAV. Effects of the chemokine CCL2 on blood-brain barrier permeability during ischemia-reperfusion injury. J Cereb Blood Flow Metab. 2006;26(6):797–810. doi: 10.1038/sj.jcbfm.9600229 .16192992

[17] McCollBW, RothwellNJ, AllanSM. Systemic inflammation alters the kinetics of cerebrovascular tight junction disruption after experimental stroke in mice. J Neurosci. 2008;28(38):9451–62. doi: 10.1523/JNEUROSCI.2674-08.2008 18799677PMC6671112

[18] AbdullahiW, TripathiD, RonaldsonPT. Blood-brain barrier dysfunction in ischemic stroke: targeting tight junctions and transporters for vascular protection. American journal of physiology Cell physiology. 2018;315(3):C343–C56. doi: 10.1152/ajpcell.00095.2018 29949404PMC6171039

[19] BedersonJB, PittsLH, TsujiM, NishimuraMC, DavisRL, BartkowskiH. Rat middle cerebral artery occlusion: evaluation of the model and development of a neurologic examination. Stroke. 1986;17(3):472–6. doi: 10.1161/01.str.17.3.472 .3715945

[20] CheslowL, AlvarezJI. Glial-endothelial crosstalk regulates blood-brain barrier function. Curr Opin Pharmacol. 2016;26:39–46. doi: 10.1016/j.coph.2015.09.010 .26480201

[21] EltzschigHK, EckleT. Ischemia and reperfusion—from mechanism to translation. Nat Med. 2011;17(11):1391–401. doi: 10.1038/nm.2507 22064429PMC3886192

[22] MichalskiD, GroscheJ, PelzJ, SchneiderD, WeiseC, BauerU, et al. A novel quantification of blood-brain barrier damage and histochemical typing after embolic stroke in rats. Brain Res. 2010;1359:186–200. doi: 10.1016/j.brainres.2010.08.045 .20732314

[23] AkiguchiI, TomimotoH, SuenagaT, WakitaH, BudkaH. Blood-brain barrier dysfunction in Binswanger’s disease; an immunohistochemical study. Acta Neuropathol. 1998;95(1):78–84. doi: 10.1007/s004010050768 .9452825

[24] ChenJ, JinH, XuH, PengY, JieL, XuD, et al. The Neuroprotective Effects of Necrostatin-1 on Subarachnoid Hemorrhage in Rats Are Possibly Mediated by Preventing Blood-Brain Barrier Disruption and RIP3-Mediated Necroptosis. Cell Transplant. 2019;28(11):1358–72. doi: 10.1177/0963689719867285 31370690PMC6802141

[25] RehorovaM, VargovaI, ForostyakS, VackovaI, TurnovcovaK, Kupcova SkalnikovaH, et al. A Combination of Intrathecal and Intramuscular Application of Human Mesenchymal Stem Cells Partly Reduces the Activation of Necroptosis in the Spinal Cord of SOD1(G93A) Rats. Stem Cells Transl Med. 2019;8(6):535–47. doi: 10.1002/sctm.18-0223 30802001PMC6525562

[26] NaitoH, NojimaT, FujisakiN, TsukaharaK, YamamotoH, YamadaT, et al. Therapeutic strategies for ischemia reperfusion injury in emergency medicine. Acute Med Surg. 2020;7(1):e501. doi: 10.1002/ams2.501 32431842PMC7231568

[27] ChenAQ, FangZ, ChenXL, YangS, ZhouYF, MaoL, et al. Microglia-derived TNF-alpha mediates endothelial necroptosis aggravating blood brain-barrier disruption after ischemic stroke. Cell death & disease. 2019;10(7):487. doi: 10.1038/s41419-019-1716-9 31221990PMC6586814

[28] DegterevA, OfengeimD, YuanJ. Targeting RIPK1 for the treatment of human diseases. Proceedings of the National Academy of Sciences of the United States of America. 2019;116(20):9714–22. doi: 10.1073/pnas.1901179116 31048504PMC6525537

[29] WangYQ, WangL, ZhangMY, WangT, BaoHJ, LiuWL, et al. Necrostatin-1 suppresses autophagy and apoptosis in mice traumatic brain injury model. Neurochem Res. 2012;37(9):1849–58. doi: 10.1007/s11064-012-0791-4 .22736198

[30] NewtonK, DuggerDL, MaltzmanA, GreveJM, HedehusM, Martin-McNultyB, et al. RIPK3 deficiency or catalytically inactive RIPK1 provides greater benefit than MLKL deficiency in mouse models of inflammation and tissue injury. Cell death and differentiation. 2016;23(9):1565–76. doi: 10.1038/cdd.2016.46 27177019PMC5072432

[31] QuY, TangJ, WangH, LiS, ZhaoF, ZhangL, et al. RIPK3 interactions with MLKL and CaMKII mediate oligodendrocytes death in the developing brain. Cell death & disease. 2017;8(2):e2629. doi: 10.1038/cddis.2017.54 28230861PMC5386494

[32] ChenH, FangY, WuJ, ChenH, ZouZ, ZhangX, et al. RIPK3-MLKL-mediated necroinflammation contributes to AKI progression to CKD. Cell death & disease. 2018;9(9):878. doi: 10.1038/s41419-018-0936-8 30158627PMC6115414

[33] ZhuH, SunA. Programmed necrosis in heart disease: Molecular mechanisms and clinical implications. J Mol Cell Cardiol. 2018;116:125–34. doi: 10.1016/j.yjmcc.2018.01.018 .29426003

[34] HribljanV, LisjakD, PetrovicDJ, MitrecicD. Necroptosis is one of the modalities of cell death accompanying ischemic brain stroke: from pathogenesis to therapeutic possibilities. Croat Med J. 2019;60(2):121–6. doi: 10.3325/cmj.2019.60.121 31044583PMC6509625

[35] ItoY, OfengeimD, NajafovA, DasS, SaberiS, LiY, et al. RIPK1 mediates axonal degeneration by promoting inflammation and necroptosis in ALS. Science. 2016;353(6299):603–8. doi: 10.1126/science.aaf6803 27493188PMC5444917

[36] OfengeimD, YuanJY. Regulation of RIP1 kinase signalling at the crossroads of inflammation and cell death. Nat Rev Mol Cell Bio. 2013;14(11):727–36. doi: 10.1038/nrm3683 24129419

[37] AminP, FlorezM, NajafovA, PanH, GengJ, OfengeimD, et al. Regulation of a distinct activated RIPK1 intermediate bridging complex I and complex II in TNFalpha-mediated apoptosis. Proceedings of the National Academy of Sciences of the United States of America. 2018;115(26):E5944–E53. doi: 10.1073/pnas.1806973115 29891719PMC6042106

[38] WallachD, KangTB, DillonCP, GreenDR. Programmed necrosis in inflammation: Toward identification of the effector molecules. Science. 2016;352(6281). doi: 10.1126/science.aaf2154 27034377

[39] SunLM, WangHY, WangZG, HeSD, ChenS, LiaoDH, et al. Mixed Lineage Kinase Domain-like Protein Mediates Necrosis Signaling Downstream of RIP3 Kinase. Cell. 2012;148(1–2):213–27. doi: 10.1016/j.cell.2011.11.031 22265413

[40] OfengeimD, ItoY, NajafovA, ZhangY, ShanB, DeWittJP, et al. Activation of necroptosis in multiple sclerosis. Cell Rep. 2015;10(11):1836–49. doi: 10.1016/j.celrep.2015.02.051 25801023PMC4494996

[41] LiuC, FuQ, MuR, WangF, ZhouC, ZhangL, et al. Dexmedetomidine alleviates cerebral ischemia-reperfusion injury by inhibiting endoplasmic reticulum stress dependent apoptosis through the PERK-CHOP-Caspase-11 pathway. Brain Res. 2018;1701:246–54. doi: 10.1016/j.brainres.2018.09.007 .30201260

[42] LiuZ, LiuY, ZhouH, FuX, HuG. Epoxyeicosatrienoic acid ameliorates cerebral ischemia-reperfusion injury by inhibiting inflammatory factors and pannexin-1. Mol Med Rep. 2017;16(2):2179–84. doi: 10.3892/mmr.2017.6831 .28656267

[43] NorstedE, GomucB, MeisterB. Protein components of the blood-brain barrier (BBB) in the mediobasal hypothalamus. J Chem Neuroanat. 2008;36(2):107–21. doi: 10.1016/j.jchemneu.2008.06.002 .18602987

[44] HaraH, HuangPL, PanahianN, FishmanMC, MoskowitzMA. Reduced brain edema and infarction volume in mice lacking the neuronal isoform of nitric oxide synthase after transient MCA occlusion. J Cereb Blood Flow Metab. 1996;16(4):605–11. doi: 10.1097/00004647-199607000-00010 .8964799

[45] JuF, RanY, ZhuL, ChengX, GaoH, XiX, et al. Increased BBB Permeability Enhances Activation of Microglia and Exacerbates Loss of Dendritic Spines After Transient Global Cerebral Ischemia. Front Cell Neurosci. 2018;12:236. doi: 10.3389/fncel.2018.00236 30123113PMC6085918

[46] TuYF, TsaiYS, WangLW, WuHC, HuangCC, HoCJ. Overweight worsens apoptosis, neuroinflammation and blood-brain barrier damage after hypoxic ischemia in neonatal brain through JNK hyperactivation. J Neuroinflammation. 2011;8:40. doi: 10.1186/1742-2094-8-40 21518436PMC3090337

[47] JaattelaM, MouritzenH, EllingF, BastholmL. A20 zinc finger protein inhibits TNF and IL-1 signaling. Journal of immunology. 1996;156(3):1166–73. .8557994

[48] MalewiczM, ZellerN, YilmazZB, WeihF. NF kappa B controls the balance between Fas and tumor necrosis factor cell death pathways during T cell receptor-induced apoptosis via the expression of its target gene A20. The Journal of biological chemistry. 2003;278(35):32825–33. doi: 10.1074/jbc.M304000200 .12813034

